# A Hypercoagulable Hematological Metastasis Breast Cancer Model

**DOI:** 10.1155/2021/5473959

**Published:** 2021-08-26

**Authors:** Wen-Jing Yang, Gan-Lin Zhang, Ke-Xin Cao, Guo-Wang Yang

**Affiliations:** Department of Oncology, Beijing Hospital of Traditional Chinese Medicine, Capital Medical University, Beijing 100010, China

## Abstract

**Background:**

The hypercoagulable status, which forms a vicious cycle with hematogenous metastasis, is a common systemic alteration in cancers. As modeling is a key approach in research, a model which is suitable for studying how the hypercoagulable status promotes hematogenous metastasis in breast cancer is urgently needed.

**Methods:**

Based on the tumor-bearing period (TBP) and postoperative incubation period (PIP), 4T1-breast cancer models were constructed to evaluate coagulation and tumor burden to generate multiple linear regression-based lung metastasis prediction formula. Platelets and 4T1 cells were cocultured for 30 min or 24 h *in vitro* to evaluate the early and late phases of their crosstalk, and then the physical characteristics (concentration and size) and procoagulant activity of the coculture supernatants were assayed.

**Results:**

The multiple linear regression model was constructed as log10 (photon number) = 0.147 TBP + 0.14 PIP + 3.303 (TBP ≤ 25 and PIP ≤ 17) to predict lung metastasis. Coculture of platelets and 4T1 cells contributed to the release of extracellular vesicles (EVs) and the development of the hypercoagulable status.

**Conclusions:**

*In vivo* and *in vitro* hypercoagulable status models were developed to explore the mechanism of hypercoagulable status which is characterized by platelet activation and promotes hematogenous metastasis in breast cancer.

## 1. Introduction

The hypercoagulable status is closely related to metastasis and a poor prognosis in cancer patients [1–5]. In addition, platelet activation and aggregation and increased platelet counts have been reported to contribute to the hypercoagulable status in cancer patients [6–9]. However, reducing the number of platelets or effectively inhibiting their activation can control metastasis in experimental animal models [6–10, 11]. In addition, low-dose aspirin, which can inhibit the aggregation of platelets effectively, is recommended for primary prevention of cancer [12–16]. All the above evidence indicates that platelets play vital roles in the hypercoagulable status and tumor metastasis.

Breast cancer is the most prevalent malignant cancer that poses a serious threat to women's health worldwide. Accumulated research shows that hypercoagulability is a common complication of breast cancer and forms a vicious cycle with hematogenous metastasis [17].

Retrospective analysis of clinical data at our hospital showed that the hypercoagulable status, which is characterized by platelet activation, mainly occurred in patients with breast cancer metastasis. Currently, the relevant mechanistic studies indicate that procoagulant microparticles (MPS) with tissue factor (TF) or phospholipid (PS) expression, which come from tumor cells, platelets, or both [18–21], contribute to the hypercoagulable status and metastasis in breast cancer. EVs, including exosomes, microvesicles (MVs), and MPS [22–24], that participate in the transformation, invasion growth, hypercoagulable status, and drug-resistance of cancer cells have been recognized as critical mediators of extracellular communication. PS exposed on EVs has been widely reported to promote the hypercoagulable status and metastasis in breast cancer [25–27]. However, the mechanism of EVs in hypercoagulable status to promote the progression in breast cancer has not been fully revealed.

Given the mechanism underlying the hypercoagulable status, which is characterized by platelet activation and contributes to breast cancer metastasis, has not been fully revealed. As an efficient and stable model is recognized as a key basis for research [28], which is contributed to explore the underlying mechanism of that, we committed to constructing *in vivo* and *in vitro* models in this field. In this study, by constructing and comprehensively evaluating the effectiveness of *in vivo* and *in vitro* models, we provide powerful research tools to study the hypercoagulable status that is characterized by platelet activation in the context of promoting hematogenous metastasis in breast cancer.

## 2. Materials and Methods

### 2.1. Validating the Hypercoagulable Status in Breast Cancer Patients

A retrospective analysis was performed with breast cancer patients who had undergone a TEG assay at the Beijing Traditional Chinese Medicine Hospital, Capital Medical University between July 2016 and May 2019. Clinical information (pathological diagnosis, clinical stage, combined disease status, medical history, sex, and age) and TEG results were obtained at the same time. The inclusion criteria were as follows: pathological diagnosis of breast cancer and completion of a TEG test. The exclusion criteria were as follows: unclear clinical staging, receipt of anticoagulant therapy within 2 weeks, receipt of radiotherapy or chemotherapy within 1 month, and the presence of coagulation-related diseases.

The TEG parameters included *R* (min), *K* (min), angle (deg), and MA (mm). *R* reflects the prothrombin initiation time, with a prolonged *R* indicating a lack of coagulation factors and a shortened *R* indicating that the blood is hypercoagulability. MA reflects the maximum activity of platelets, with an increased MA indicating hypercoagulability and a reduced MA indicating platelet dysfunction.

### 2.2. Cell Culture

The murine breast cancer 4T1/4T1-luc cell line was obtained from the Shanghai Institute of Cell Biology, Chinese Academy of Sciences. The 4T1/4T1-luc cell line was cultured in RPMI-1640 medium (Sigma-Aldrich, USA) supplemented with 10% fetal bovine serum (FBS; Sigma-Aldrich, USA) and 1% penicillin streptomycin (Gibco; 10000 units/ml penicillin and 10000 *μ*g/ml streptomycin) in a humidified atmosphere (5% CO2, 37°C).

### 2.3. Animal Care

6-8-week-old female BALB/c mice were obtained from Beijing Vital River Laboratory Animal Technology Co. Ltd., and animal protocols were approved by the China Laboratory Animal Welfare and Animal Experimental Ethical Committee (2018030209). All mice were maintained in specific pathogen-free barrier facilities at the Beijing Institute of Traditional Chinese Medicine, carefully bred, and humanely sacrificed by cervical dislocation after anesthesia administration at the study endpoint.

### 2.4. 4T1-Luc Lung Metastasis Model Establishment

On the basis of a previous study [29, 30], 4T1-luc cells were harvested and suspended at the concentration of 2 × 10^7^/mL in PBS. Then, 50 *μ*l cell suspension (1 × 10^6^) was steadily injected into the fourth intramammary gland fat pad of female BALB/c mouse at a consistent speed. According to our experience on the regularity of lung metastasis, the TBP and PIP are both important in lung metastasis, and 20 days ± 2 days is nearly the lowest requirement for successful lung metastasis, 27 days ± 2 days is nearly the longest time for control the volume of the breast tumor so as not to affect the free movement of mice. In addition, 15 days ± 2 days or 1 day were additionally time for circulating breast tumor cells successfully metastasize and grow in the lung. Therefore, four experimental groups based on these parameters were set up. According to the TBP, the mice were divided into two groups (27 days ± 2 days and 20 days ± 2 days). According to the PIP (15 days ± 2 days, 1 day), the two groups were further divided into 4 total subgroups: TBP 25 + PIP 17, TBP 29 + PIP 1, TBP 22 + PIP 13, and TBP 18 + PIP 1. A normal group was also set up.

According to the TBP, breast tumors were removed as follows: first, a mouse was fixed on a paraffin table in the supine position with inhaled anesthesia (oxygen : isoflurane = 98 : 2). Next, importantly, the mouse was disinfected with 70% alcohol, and ophthalmic forceps were used to lift the upper right corner of the tumor, which was removed carefully with surgical scissors from the left side of the mammary fat pad. According to the radical principle, tumor-free principle, and aseptic principle, attention was paid to clearly detach the blood vessels, completely eliminate the tumor capsule, and thoroughly disinfect the work space and animal, respectively. Notably, complete separation and proximal ligation of the main nutrient vessel were key to reducing bleeding (Figure 1). Ultimately, the incision was sutured closed using 5-0 nonabsorbable surgical sutures, and the animals were observed daily.

### 2.5. Evaluation of the *In Vivo* Model

#### 2.5.1. Evaluation of Breast Tumor

Beginning on the 10th day after modeling, tumor form and volume were recorded every 3 days. Tumor volume (*V*) was calculated with the formula: *V* (mm^3^) = 0.5 × *a* × *b*^2^ (*a* = the shortest diameter, and *b* = the longest diameter).

After breast tumor weight was measured and photos were taken, the tumors were immersion-fixed in 10% neutral buffered formalin for 24 h and processed for paraffin embedding. Paraffin blocks of tumor tissue were prepared to 5 *μ*m sections and stained with H&E.

#### 2.5.2. Evaluation of Lung Metastasis

Before sacrifice, the pulmonary and extrapulmonary metastatic lesions of mice were assessed by optical *in vivo* imaging (IVIS-Lumina III). The specific protocol was as follows: mice were injected subcutaneously with 200 *μ*l fluorescein substrates, anesthetized with isoflurane for 3 min, placed into a live fluorescence imaging system, and finally analyzed with Living Image 4.5 software. The pathological confirmation method for the pulmonary and extrapulmonary metastatic lesions was the same as that used for the breast tumors.

#### 2.5.3. Evaluation of Animal Welfare/Surgical Feasibility

According to the principle of animal welfare, we evaluated our model from the following aspects: (1) total time spent to remove the breast tumor, with the expectation that the shorter the time, the less harmful the procedure was to the mouse; (2) the length of the breast surgical incision, with the expectation that the shorter the incision, the less harmful the procedure was to the animal; and (3) the trend in animal weight variation, with the expectation that the milder the trend, the less harmful the procedure was to the animal.

#### 2.5.4. TEG Assay

BALB/c mouse whole blood (500 *μ*l) was anticoagulated with 3.8% sodium citrate. The analysis was performed as follows: the instrument was calibrated, 20 *μ*l calcium chloride was pushed to the bottom of the test cup, the 500 *μ*l anticoagulant-treated blood was mixed with 20 *μ*l kaolin thoroughly to stimulate the blood, 360 *μ*l stimulated blood was transferred to the TEG test cup, and then testing was started.

### 2.6. 4T1 Cell and Platelet Coculture Model Establishment [29–31]

#### 2.6.1. Preparation of Mouse Platelets

Blood samples were obtained from female BALB/c mice. Washed platelet suspensions were prepared from the blood in Tyrode's solution as previously described (1 × 10^8^/ml) and then suspended in RPMI-1640 medium (1 × 10^8^/ml).

#### 2.6.2. Establishment of the *In Vitro* Model

To study the crosstalk between platelets and breast tumor cells in cancer progression, BALB/c mouse platelets and 4T1 cells were cultured together to obtain the coculture supernatants. Under physiological conditions, the lifespan of platelets is 7-10 days. However, *in vitro*, that survival time was greatly shortened. We defined the *in vitro* culture time of 30 min to mimic the early-phase crosstalk that occurs *in vivo* and the *in vitro* culture time of 24 h to mimic the late-phase crosstalk *in vivo*. 4T1 cells in the log phase were harvested and counted, and then the concentration was adjusted to 1 × 10^6^/mL with RPMI-1640 medium. Warmed 25 mM Cacl_2_ (1 *μ*l) was added before washed platelet suspensions (1 ml), and 4T1 cell suspensions (1 ml) were cocultured (37°C, 5% CO2). At the defined endpoints, the coculture supernatants were centrifuged twice (1400 × g for 20 min and then 13000 × g for 2 min) at 4°C to remove all of the 4T1 cells and platelets completely. Platelets/4T1 cells were also cultured separately for 30 min or 24 h as independent controls, and the supernatants were stored at -80°C until assayed.

In addition, to validate if the trend in 4T1 mouse mammary tumor cells and BALB/c mouse platelets was also observed with human breast cancer cells and human platelets, we used MDA-MB-231 human breast cancer cells and human platelets to repeat the validation test.

### 2.7. Identification of the Coculture Supernatants

#### 2.7.1. Physical Characteristics (Concentration and Size)

Supernatants were analyzed with a nanoflow cytometer (N30 Nanoflow Analyzer, NanoFCM Inc, Xiamen, China), which could sensitively and rapidly perform quantitative multiparameter surface-protein profiling and sizing of individual EVs down to 40 nm.

#### 2.7.2. Procoagulant Activity

Phosphatidylserine (PS) is externalized to the outer membrane during activation or apoptosis and enhances procoagulant activity. Circulating EVs and exposed PS on different cells contribute to the procoagulant activity in patients with cancer. The procoagulant activity of supernatants was evaluated by assessing the PS exposure and Annexin V expression (Annexin V-FITC Apoptosis detection Kit, C1062).

### 2.8. Statistical Analysis

Statistical data were evaluated using SPSS 19.0 (IBM Corp. Armonk, NY, USA) and Graphpad Prim7 (Graphpad Software, Inc., USA). The specific statistical methods were the *χ*^2^, *t*-test, and one-way analysis of variance (ANOVA), *P* value < 0.05 was considered statistically significant. A multiple linear regression model was constructed to evaluate the associations of the TBP and PIP with lung metastasis.

## 3. Results

### 3.1. The Hypercoagulable Status Characterized by Platelet Activation Was Mainly Found in Patients with Metastasis

Currently, research on the hypercoagulable status of cancer patients is mainly focused on coagulation factors and platelet activation. In this study, we compared the differences in *R* and MA between patients without metastasis (*M*0) and those with metastasis (*M*1). On the one hand, the type of the hypercoagulable status of breast cancer patients was determined. On the other hand, the relationship between the hypercoagulable status and metastasis was explored. According to the inclusion and exclusion criteria, 63 women subjects were enrolled. The clinical characteristics of the eligible subjects (age 34-88 years) were as follows: 43 patients with *M*0 disease and 39 patients with *M*1 disease.

#### 3.1.1. *R* (min)

*R* < 5 indicates the hypercoagulable status (coagulation factors). The numbers of patients with the hypercoagulable status in the *M*0 and *M*1 groups were 24 and 19, respectively. In addition, the numbers of patients without the hypercoagulable status in the *M*0 and *M*1 groups were 9 and 12, respectively. There was no significant difference in *R* between the *M*0 and *M*1 groups (*χ*^2^ = 0.64, *P* > 0.05).

#### 3.1.2. MA (mm)

MA > 70 indicates the hypercoagulable status (platelets). The numbers of patients with the hypercoagulable status in the *M*0 and *M*1 groups were 0 and 5, respectively. In addition, the numbers of patients without the hypercoagulable status in the *M*0 and *M*1 groups were 33 and 25, respectively. There was a significant difference in MA between the *M*0 and *M*1 groups (*χ*^2^ = 3.91, 0.01 < *P* < 0.05).

### 3.2. TBP Plays Decisive Roles in the Volume and Weight of Breast Tumors

Breast tumor volume and weight increased as the TBP increased in all of the experimental groups (Figures 2(a) and 2(b)). In addition, the morphology of the breast tumors was recorded from the 8th day after tumor cells were injected until the 2nd day after surgery (Figure 2(c)). In addition, the breast tumor morphologies of four experimental groups were all similarly oblate, and representative H&E images of breast tumors specimens are shown in Figure 2(d) for the four experimental groups.

### 3.3. Both the TBP and PIP Play Decisive Roles in Lung Metastasis

Lung metastasis was evaluated by both lung weight and photon numbers. For lung weight, the lung weights of the four experimental groups were significantly heavier than the weight of normal group. In addition, the lung weight of the TBP 25 + PIP 17 group was significantly heavier than that of the other experimental groups, the lung weight of the TBP 25 + PIP 1 group was significantly bigger than that of the TBP 20 + PIP 17 group and the TBP 20 + PIP 1 group, the lung weight of group TBP 20 + PIP 17 was significantly bigger than that of group TBP 20 + PIP 1. However, for photon numbers, the only significantly larger number was found for the TBP 25 + PIP 17 group (Figure 3(a)). H&E staining, morphological analysis, and the photon imaging of lung metastases are shown in Figure 3(b). Unexpectedly, extrapulmonary metastasis including the chest wall, subcutaneous back sites, axillary sites, inguinal sites, and the pericardium were found in the TBP 25 + PIP 1 group and validated by H&E staining (Figure 3(c)).

### 3.4. A Multiple Linear Regression Model Was Constructed from the TBP and PIP to Predict Lung Metastasis

#### 3.4.1. Evaluation of Lung Metastasis by Photon Number

Both the TBP and the PIP were entered by stepwise selection, and there was a linear relationship among the TBP, the PIP, and lung metastasis (*F* = 15.682, *P* ≤ 0.001). Both the TBP and the PIP were independent predictors of lung metastasis (*R*^2^ = 0.599, Durbin − Watson = 1.494), and a regression equation was constructed with coefficients: log_10_^(photonnumber)^ = 0.147, TBP + 0.14, PIP + 3.303, where the *P* values of the TBP, PIP, and constant were 0.010, 0.017, and ≤0.001, respectively. No obvious collinearity between the TBP (VIF = 1.000) and the PIP (VIF = 1.000) was observed. (∣Std.Residual | <3, minimum = −1.594, maximum = 2.759), but Gaussian distributions were found (Table 1).

#### 3.4.2. Evaluation of Lung Metastasis by Lung Weight

The TBP was eliminated by stepwise selection, and there was no linear relationship between the PIP and lung metastasis (*F* = 8.413, *P* = 0.08). The PIP was not useful for lung metastasis prediction (by lung weight) (*R*^2^ = 0.277, Durbin − Watson = 1.926) (Table 1).

### 3.5. An *In Vivo* Model in Which with the Hypercoagulable Status Was Characterized by Platelet Activation

There were no significant differences between the four experimental groups and the normal group in terms of *R* (min). However, there were significant differences between the four experimental groups and normal group in terms of MA (mm) (Figure 4).

### 3.6. Evaluation of Animal Welfare/Feasibility of an Operation

Operation time and incision length increased as the TBP increased. These increases undoubtedly increased animal trauma and the difficulty of the operation. The TBP 25 + PIP 17 group had the longest operation time and the longest incision length among the four experimental groups, the TBP 25 + PIP 17 group spent a longer time in surgery and had a longer incision length than the TBP20 + PIP 17 and TBP 20 + PIP 1 groups, and the TBP 20 + PIP 17 group spent a longer time in surgery and had a longer incision length than the TBP 20 + PIP 1 group (Figure 5).

### 3.7. Evaluation of Characteristics of Supernatants

Supernatants were obtained according to previously published methods [31–33]. Physical characteristics (concentration and size) of the supernatants were as follows (Table 2): (1) within a certain period of time (30 min–24 h), extension of the culture time promoted release; (2) coculture promoted release; and (3) there was no significant difference in EV size among the supernatants. In addition, the EVs with exposed PS in the 24 h coculture supernatant were significantly more numerous than those in the 24 h platelet culture supernatant (Table 3).

## 4. Discussion

Breast cancer is the most common malignant cancer in women worldwide, and metastasis seriously increases the risk of death [34, 35]. More than 60% of malignant tumor patients develop the hypercoagulable status as a complication. In addition, this status further affects metastasis, treatment strategies, and even patient prognosis. The retrospective analysis of clinical data from our hospital indicated that the hypercoagulable status characterized by platelet activation was mainly found in patients with metastasis. However, the related mechanism has not been fully revealed.

Given that an efficient and stable model is a key basis for research [28], we committed to constructing *in vivo* and *in vitro* models in this field. An “ideal model” mimics human disease as closely as possible. In addition, the rule of 3Rs (reduction, refinement, and replacement) should be kept in mind. As different researchers have different preferences for lung metastasis, we established the multiple linear regression equation (log_10_^(photonnumber)^ = 0.147 TBP + 0.14 PIP + 3.303) to predict lung metastasis. Which means researchers can achieve preferences lung metastasis by controlling TBP and PIP. In addition, we confirmed that the photon number is a more reliable predictor of lung metastasis than lung weight.

In our analysis of the decisive roles of the TBP and PIP in lung metastasis, we found that (1) when the TBP is too short, the tumor does not have time to undergo invasion and metastasis, which directly affects the success of metastasis; in contrast, when the TBP is too long, the tumor invades the surrounding tissue, which undoubtedly increases the difficulty of achieving effective surgical treatment. On the one hand, prolonged anesthesia exposure may lead to animals dying. However, incomplete resection exposure may lead to local recurrence. In conclusion, in regard to lung metastasis, the shorter the TBP is, the better. In addition, in terms of surgical techniques, we emphasize that complete separation and proximal ligation of the main nutrient vessel are key to reducing blood loss, which obviously decreases animal trauma (Figure 1). (2) For the PIP, although the TBP of the TBP 25 + PIP 17 group was shorter than that of the TBP 25 + PIP 1 group, lung metastasis was more obvious in the TBP 25 + PIP 17 group than that of the TBP 25 + PIP 1 group, and the TBP 25 + PIP 17 group even exhibited extrapulmonary metastasis. This indicated that if the TBP was over 25 days, a continued extension of the TBP did not increase the incidence of lung metastasis. In contrast, the PIP of the TBP 25 + PIP 17 group was longer than that of the TBP 20 + PIP 17 group, which indicated that when the TBP was over 22 days, a prolonged PIP could increase the incidence of extrapulmonary metastasis. This means that to establish an efficient and stable hypercoagulable status model, the TBP should be no more than 25 days, and the PIP should be no more than 17 days.

Through evaluation of the hypercoagulable status, we found that (1) compared with the normal group, all of the experimental groups showed a hypercoagulable status characterized by platelet activation, which indicated that our *in vivo* model is particularly suitable for studying the hematological metastasis mechanism underling the hypercoagulable status characterized by platelet activation in breast cancer; (2) the TBP 25 + PIP 1 group, which had the biggest MA of the four experimental groups, was characterized by the biggest TBP, indicating that the TBP might have an important influence on the activation of platelets; and (3) the TBP 20 + PIP 1 group did not develop obvious lung metastasis but exhibited the hypercoagulable status, indicating that development of hypercoagulable status in our *in vivo* model is an early event in metastasis, which effectively mimics the biological process of the hypercoagulable status promoting metastasis.

Dynamic crosstalk between tumors and platelets is recognized as a key regulator of the hypercoagulable status and malignant progression. For our research, we established an *in vitro* model by coculturing breast tumor cells (mouse/human) and platelets (mouse/human). The physical characteristics of the supernatants indicated that (1) within a certain period of culture time (30 min–24 h), extending the culture time promoted release; (2) coculture promoted release; and (3) there were no significant differences in EV size among the tested supernatants. The procoagulant activity of the supernatants indicated coculturing breast tumor cells and platelets significantly increased procoagulant activity. In addition, the coculture system was further used to validate the contributions to EV release and the hypercoagulable status in breast cancer progression.

## 5. Conclusions

The retrospective analysis of clinical data from our hospital indicated the hypercoagulable status characterized by platelet activation was mainly found in patients with metastasis. To explore the associated mechanism by modeling, since it is well known that modeling is a key basis of research, we committed to constructing model suitable for studying how the hypercoagulable status promotes hematogenous metastasis in breast cancer. *In vivo*, based on the important independent variables TBP and PIP, a multiple linear regression model was constructed to predict lung metastasis: log_10_^(photonnumber)^ = 0.147 TBP + 0.14 PIP + 3.303 (TBP ≤ 25 and PIP ≤ 17). *In vitro*, supernatants were obtained following coculture of breast tumor cells and platelets. In addition, the coculture system was further used to validate the contributions to EV release and the hypercoagulable status in breast cancer progression. In conclusion, we provided useful *in vivo* and *in vitro* hypercoagulable status models to study the mechanism of hematological metastasis in breast cancer.

## Figures and Tables

**Figure 1:** Complete separation and proximal ligation of the main nutrient vessel.

**Figure 2:** The volume, weight, morphology, and H&E staining of breast tumors. (a) The volume of the breast tumors increased as the TBP increased in all experimental groups. (b) The weight of the breast tumors increased with the TBP in all of the experimental groups. (c) The morphology of the breast tumors was recorded from the 8th day after the tumor cells were injected to the 2nd day after the surgery. (d) The morphology and H&E validation of the breast tumors in the four experimental groups are shown.

**Figure 3:** Evaluation of pulmonary and extrapulmonary metastasis. (a) The weight and photon number of lung metastases were compared among the four experimental groups. Lung metastasis is shown by lung weight and photon number. (b) The H&E staining, morphology, and photon imaging of lung metastases in the four experimental groups are shown. (c) Extrapulmonary metastasis include the chest wall, subcutaneous back sites, axillary sites, inguinal sites, and the pericardium in the TBP 25 days, PIP 17 days group, which was validated by H&E staining.

**Figure 4:** TEG analysis *R* (min) and MA (mm) parameters in the *in vivo* model. There were no significant differences between the four experimental groups and the normal group in regard to *R* (min). However, there were significant differences between the four experimental groups and the normal group for the MA (mm).

**Figure 5:** Evaluation of operation time and incision length for in the *in vivo* model: both the operation time and incision length increased as the TBP increased.

**Table 1:** The multiple linear regression model was constructed with the TBP and PIP to predict lung metastasis.

	Model^a^ (p value)	Model^b^
ANOVA(F)	15.682 (≤0.001)	8.413 (0.008)
Constant	3.303 (0.017)	145.197 (≤0.001)
PIP coefficients	0.14 (≤0.001)	5.222 (0.008)
TBP coefficients	0.147 (0.10)	
Adjusted R Square	0.561	0.244
Durbin-Watson	1.494	1.926
Std. Residual	-1.594~2.759	-1.028~3.312

a Predictors: (Constant), PIP, TBP; Dependent Variable: log_10_^(Flux)^. b Predictors: (Constant), PIP; Dependent Variable: lung weight.

**Table 2:** Physical characteristics (concentration and size) of supernatants. (1) Within a certain period of culture time (30 min-24 h), extension of the culture time promoted release. (2) Coculture promoted release. (3) There were no significant differences in EV size among the supernatants.

Sample	Size(nm)	Concentration
4T1 (30 min)	61.14 ± 16.45	5.45 × 10^9^
4T1 (24 h)	57.63 ± 16.91	9.47 × 10^9^
PLT (30 min)	64.26 ± 27.31	2.39 × 10^10^
PLT (24 h)	57.35 ± 19.73	3.28 × 10^10^
4T1+PLT (30 min)	61.79 ± 24.34	2.97 × 10^10^
4T1 + PLT (24 h)	57.37 ± 19.55	5.73 × 10^10^

4T1: murine breast cancer cell line. PLT: platelets obtained from a BALB/c mouse. 4T1 + PLT: coculture of the murine breast cancer cell line and the PLTs obtained from the BALB/c mouse.

**Table 3:** The procoagulant activity of the 24 h coculture supernatant was significantly higher than that of the 24 h platelets supernatant.

Sample	Size(nm)	Concentration
PLT (24 h)	82.36±28.29	5.84×10^9^
4T1 + PLT (24 h)	76.91±29.26	9.86×10^9^

PLT: platelets obtained from a BALB/c mouse. 4T1 + PLT: coculture of a murine breast cancer cell line and the PLTs obtained from the BALB/c mouse.

## Data Availability

All data used or analysed during this study are included in this published article.
